# A Dynamic Equilibrium Mechanism of Core Layer Interests in the Mobile Medical Platform Ecosystem

**DOI:** 10.1155/2022/8915055

**Published:** 2022-01-21

**Authors:** Zheng Shenghua, Hakam Bader, Chen Jue

**Affiliations:** ^1^School of Management, Zhejiang University of Technology, Hangzhou 310023, China; ^2^School of Tourism and Urban-Rural Planning, Zhejiang Gongshang University, Hangzhou 310018, China

## Abstract

In recent years, with the development of the mobile Internet, big data, and cloud computing, the mobile medical platforms such as Ding Xiang Yuan aggregating platform ecological resources have played an irreplaceable role in improving efficiency, optimizing resource allocation, and even promoting the transformation and upgrading of the medical industry. Despite all this, most mobile medical platforms in China still face many problems, including the immature business model, the stagnation of the interaction of knowledge and information among platform members, and the weak platform competitiveness. Based on a review of the platform and commercial ecosystems, this paper adopts the evolutionary game method and simulation to analyze the evolutionary stability strategy of operators, partners, and users in the core layer of the platform during preflow and postflow periods of a mobile medical platform, hence, to construct a beneficial dynamic equilibrium model of a platform business ecosystem under the optimal decisions made by all parties involved in the platform: the goal in the early stage (preflow period) is to increase platform user flow. Hence, the knowledge/information sharing of platform users is needed to enhance platform's visibility. While in the late period (postflow period), when the platform user flow reaches a certain scale, platform's goal is to promote revenue, which relies mainly on the pricing strategy. It is critical to promote the stability of the platform and the dynamic balance of interests at the core layer in the pricing process. This paper applies the platform business ecosystem theory and the evolutionary game theory to mobile medical platform development, contributing theoretically and practically in the following: (1) providing a more solid theoretical support for the mobile medical platform research and enriching the theoretical framework of the platform business ecosystem; (2) proposing the dynamic equilibrium model based on the optimal decisions of the platform core layers, which help to reveal the inherent law of the evolution of the mobile medical platform; (3) providing policy suggestions and management implications in constructing an appropriate business ecosystem and achieving sustainable development in mobile medical platforms.

## 1. Introduction

The mobile medical platform is an emerging medical service format, which uses mobile Internet as the carrier and uses big data, wearable devices, and cloud computing as the means [1]. Integrating the supply of diagnosis and treatment services, the allocation of medical resources, and the configuration of all-factor links in medical insurance, a mobile medical platform can provide online and offline closed-loop services [2]. By means of patient-driven operations, medical institution efficiency improvement, and “sinking” high-quality medical resources, the mobile medical platform, having a subversive impact on the traditional medical service model, overcomes many shortcomings in traditional services including the uneven distribution and inefficient use of traditional medical resources, poor information sharing, and poor user experience [3, 4]. Accordingly, the Chinese government has successively promulgated many important policies, such as the “Guiding Opinions on Actively Promoting ‘Internet +' Actions” and the “Outline of ‘Healthy China 2030'.” The provision of “Internet + Medical” services has become an important part of the national “Internet +” strategy. Driven by internal and external factors, mobile medical platforms, such as Ding Xiang Yuan, Micro-Medicine, and Ali Health, are experiencing an explosive growth. By the end of 2017, there were 36 mobile medical platforms with more than 300 million users in China [3]. The investment in mobile medical platforms was estimated to be approximately 14 billion yuan [2] at the end of 2018. The mobile medical platform is becoming an innovative solution to the medical difficulties of 1.3 billion Chinese people, bringing tremendous value to hospital systems, patients, and government supervision, and could contribute to the development of the medical sector in the rest of the world.

However, as a new form of medical organization, the mobile medical platform has also encountered many bottlenecks in its rapid growth. Firstly, relevant regulations and policies (e.g., industry entrance permission, qualification verification) and related supervision at the national level are inadequate; secondly, the platform structure remains imperfect, causing asymmetric information between doctors and patients and a low participation rate among doctors [5]; thirdly, industry chain is incomplete, bringing low user awareness of the platform and weak user stickiness and low utilization of user data; fourthly, the business model is still immature together with the low level of integration and imperfect service functions [2, 3]. As a result, the platform could not attract enough users in the early stage and turn the user flows into revenue in the later stage, reducing the sustainability of the platform.

These problems are due to the fact that the mobile medical platform is essentially a platform business ecosystem composed of platform operators, suppliers (doctors), and demanders (patients) [6, 7], and its operation effectiveness depends on a resource matching between supply and demand and the dynamic balancing of the interests among the platform participants. Therefore, how to achieve the supply-demand matching in resources and the dynamic evolutionary equilibrium of all platform participants to facilitate the sustainable development of the mobile medical platform has become an urgent problem for which solutions have been examined in both theoretical and industrial circles.

Based on this understanding, this paper applies the platform business ecosystem theory and the evolutionary game theory into the research of mobile medical platform development, intending thereby to make the following theoretical and practical contributions: (1) providing a more solid theoretical support for the research of the mobile medical platform, this paper tries to enrich and improve the theoretical framework of the platform business ecosystem. (2) To reveal the inherent law of the evolution of mobile medical platform, based on the optimal decisions of the platform core layer, this study proposes the dynamic equilibrium model to analyse the interests of the platform business ecosystem.

## 2. Literature Review

### 2.1. Research on Mobile Medical

In 2002, a study published by Price and Summers [1], Clinical Knowledge Management and M-health, explored for the first time the relationship between mobile medical communication equipment and clinical knowledge management [4, 8]. Mobile Health was defined as the use of mobile communication tools to provide medical services and information, such as remote patient monitoring, online consultation, personal care equipment, and wireless access to electronic medical records and prescriptions [1, 9]. The information distribution usually comprises the B2B mode, which is based on activities such as communication among medical workers, knowledge sharing and the application of medical tools, and the B2C mode, which is based on activities such as online appointment registration, consultation, and medical record inquiry [10, 11]. Showing great potential for development, mobile health has benefited from the maturity of the national medical reform policy, the improvement of living standards, the renewal of life concepts, the transformation of Internet technology, and the shortage and unreasonable distribution of medical resources [8]. At the same time, a variety of inherent innovations have enabled mobile medical operations to be distributed closer and closer to the areas where services are required [12]. At the technical level, using smartphones to collect and analyse patient data improves the process of convenient collection, rapid transmission, and the intelligent analysis of patient data. In addition, the deep integration of the Internet of Things technology and medical treatment can achieve the rapid circulation of medical information and the sharing of medical resources [13, 14]. At the market level, according to the access path of netizens' search information, we can understand their potential needs and improve existing mobile medical technology and products accordingly. At the operational level, the improvement of collaborative efficiency in the mobile medical industry chain's leading links, such as logistics, e-commerce, and online payment, is conducive to the realization of telemedicine [15, 16]. At the experience level, a mobile medical platform establishes and strengthens the trust relationship between doctors and patients, increases the supply of high-quality services, improves the service experience, and increases the user stickiness [17]. At the profit level, direct charges, transfer payments, and circular subsidies are the main sources of income [7]. At the regulatory level, assessment procedures consisting of planning and review, literature research, literature assessment, data analysis, and regular reporting effectively monitor the implementation of mobile health. More importantly, relying on the Internet integration platform, medical resources will be pooled to form a large-scale, systematic service network similar to the framework of hospitals, thereby achieving a deep crossintegration of hardware, software, and other factors [18]. As a result, the focus of mobile medical research has shifted to the platform-based mobile medical field, and the topic of discussion has begun to focus on how to integrate various factors and how to promote the development of mobile medical platforms by coordinating the relationship between the participants [1].

### 2.2. Research on the Platform

#### 2.2.1. Platform Connotation and Characteristics

A platform is an institutional arrangement form that integrates two or more distinct but interdependent interest groups to provide common solutions [8] to improve the value of the network [5, 9, 19]. A platform behaves as a kind of real or virtual space, which is externalized as products, services, and technologies and used to coordinate bilateral or multilateral trading relationships [20, 21]. The core feature of the platform is the network effect of positive externalities [22, 23]. The network effects includes the direct network effect, in which the utility of the platform to users depends on the number of platform users [24], and the indirect network effect, in which the utility of the platform to one user group depends on the number of users in another user group. A platform with more users will provide more diversified products and services [25]. Under certain conditions, a strong network effect will lead to a “winner-take-all” competition between platforms [10].

### 2.3. Platform Framework and Business Model

The network effect of the platform determines the nature of the business model of the platform characterized with “winner-take-all.” The “winner-take-all” business model [26] needs to be compatible with the economic time-space and physical space-time analysis. In these analyses, value cocreation under “Value net +” is the foundation, and following the system paradigm of the “circular industrial chain,” which involves information exchange, product sales, advertising, and other modes, the profit model is the core of the platform business model [11]. Since the users prefer value-for-money platforms, the platforms should well plan the costs and profit level. In the early stages of a platform's deployment, the subsidy strategy can be used to attract users, and in the later stage, profit can possibly be achieved based on the large-volume users.

The success of the platform business model relies on a reasonable architecture. The platform architecture is rooted in Simon's early work on a “complex system.” It consists of a set of components, interfaces between components and design rules. A system is made up of the core and peripheral components, which complement each other and are connected with each other through interfaces [13]. The platform architecture is externalized into a platform architecture layer and a user requirement layer. The former is provided by platform operating enterprises, and the latter is composed of buyer users and seller users (complementary suppliers) [14].

### 2.4. Research on Platform Business Ecosystem

A platform business ecosystem is an interdependent, dynamic interest-linking business ecosystem, which is supported by Internet technology and built around the platform to connect suppliers, distributors, complementary suppliers, end customers, and other members [16]. The technical architecture defined by the core enterprise is the foundation of the platform business ecosystem [8]. Therefore, the main structure of the platform business ecosystem (Figure 1) and its dynamic equilibrium mechanism has become the core task and focus to promote the evolution of the platform business ecosystem. Since the platform business ecosystem is affected by different combinations of interests and competition mechanisms at different evolution states, namely, the start, expansion, and maturity of the platform, the interest mechanism, that is, the interest-based game of platform's core layer is the driving force for the evolution of the platform business ecosystem.

### 2.5. Literature Enlightenment

The mobile medical platform is a typical platform business ecosystem, which is divided into a core layer and a peripheral layer (Figure 2). Among them, the core layer is composed of platform operators, partners (hospitals, doctors, pharmaceutical companies, equipment providers, etc.), and end users (patients, elderly people and groups concerned about their own health, etc.). In addition, the peripheral layer, which includes governments, intermediaries, and other stakeholders [17], works through the core layer (Figure 3). The matching of resources' supply and demand and the dynamic balancing of the interests among platform operators, partners, and end users at the core layer [4] are the core issues that must be addressed to solve the successful evolution of the mobile medical platform ecosystem.

## 3. Establishment of a Two-Stage Game Model for the Dynamic Equilibrium of Interests at the Core Layer of a Mobile Medical Platform Business Ecosystem

The mobile medical platform follows the common evolutionary characteristics and the mechanisms of a platform business ecosystem and has its own uniqueness. On the one hand, the operation of a mobile medical platform must rely on the scale of the user flow and requires professional knowledge to attract a user flow; on the other hand, the flow realization and profit model are the key to the development of the mobile medical platform. Business partners, such as hospitals, doctors, and equipment providers, are attracted to the platform and try to generate orders after obtaining the user flow. The end users who purchase the goods increase the turnover and profits of the merchants, while adding commercial value to the platform. In this way, platforms, partners, and end users become interdependent, thereby achieving the purpose of flow realization. Therefore, in view of the important role of the user flow in the dynamic equilibrium of interests at the core layer of the mobile medical platform business ecosystem and consistent with the life cycle theory of a platform business ecosystem, this paper divides the dynamic equilibrium of interests at the core layer into a preflow period, which includes a naive period and a growth period, and a postflow period, which includes a maturity period and a recession period. Based on this, this paper intends to establish the following two-stage game model: first, in the preflow period, in order to achieve the goal of increasing platform flow, the knowledge/information sharing of platform users is needed to enhance the visibility of the platform, thus promoting the increase of the platform flow. Second, in the posttraffic period, the platform flow reaches a certain scale. The goal of the platform is to promote the increase of revenue, the key to which is to solve the pricing problem. In addition, it is necessary to promote the stability of the platform and the dynamic balance of interests at the core layer in the pricing process.

### 3.1. Preflow Stage: Information Exchange Stage

#### 3.1.1. One-Time Game

*(1) Basic Assumption*. In the preflow period, the purpose of the platform is to increase the platform flow, and the two participants who promote the flow growth are the platform operators and the users. It is assumed that both of them are fully rational thinkers in terms of solving problems and are not subject to external conditions and the environment when making choices. For the knowledge possessed, the platform operators and users participating in the game can make two kinds of decision-making judgements, namely, sharing and nonsharing. The parameter description of the game is shown in Table 1; then, the game payment matrix in Table 2 can be obtained.

#### 3.1.2. Model Analysis

Through the payment matrix, it can be seen that when both sides of the game are closed and do not share knowledge and information, the profit of the final two participants is the least: the platform operator's gain is only the increase in the platform flow *f*_2_, while the end user's gain is the improvement in self-efficacy *e*_2_. In addition, the profit is *f*_2_ − *o*_2_ and *e*_2_ − *c*_2_. If only the platform operator chooses the sharing strategy in the game, then he or she will obtain more profits than that obtainable through the nonsharing strategy: in addition to the increase in platform flow, the platform operator will obtain the profits brought by the improvement of platform's competitiveness and information capability; however, he or she will also need to pay more operating costs. In this case, the benefits of the platform and the users are denoted by *f*_1_ + *a*_0_ + *t*_0_ − *o*_1_ and *e*_2_ − *c*_2_. Similarly, if only the platform user chooses the sharing strategy, he or she will obtain more profits than that obtainable through the nonsharing strategy: the knowledge ability and the platform identity of end users will be improved, and the benefits of both are denoted by *f*_2_ − *o*_2_ and *e*_1_ + *k*_0_ + *i*_0_ − *c*_1_. If both parties choose the sharing strategy, they will obtain an extra benefit. The extra benefit of the platform operator is *α*_1_, and the extra benefit of the platform user is *α*_2_; then, the benefits of both are *f*_1_ + *a*_0_ + *t*_0_ + *α*_1_ − *o*_1_ and *e*_1_ + *k*_0_ + *i*_0_ + *α*_2_ − *c*_1_. Similarly, the platform operators and users are analysed for strategy selection. According to the actual situation, when users choose the sharing strategy, they can obtain more desired information and a greater self-efficacy improvement. Therefore, the platform flow increases less when there is no sharing; i.e., e_1_ > e_2_ and *f*_2_ < *f*_1_. Thus, the results that can be obtained are as follows.

There are three alternative strategy combinations for the platform operator: sharing–sharing, sharing–nonsharing, and nonsharing–nonsharing. At this time, the benefit of the platform operators is *f*_1_ + *a*_0_ + *t*_0_ + *α*_1_ − *o*_0_, *f*_1_ + *a*_0_ + *t*_0_ − *o*_0_, and *f*_2_. In the case of low operating costs and high profits when sharing knowledge/information, obviously, *f*_1_ + *a*_0_ + *t*_0_ + *α*_1_ − *o*_0_ > *f*_1_ + *a*_0_ + *t*_0_ + *α*_1_ − *o*_0_ > *f*_2_; therefore, a sharing–sharing strategy is the optimal strategy for platform operators. However, if the operating cost of sharing is high, it can offset the profits or create a negative benefit; that is, *f*_2_ > *f*_1_ + *a*_0_ + *t*_0_ + *α*_1_ − *o*_0_. In this case, a nonsharing–nonsharing strategy is the optimal strategy for the platform operators.

Likewise, there are three strategy combinations for platform users to choose, namely, sharing–sharing, sharing–nonsharing, and nonsharing–nonsharing, and the corresponding benefits are *e*_1_ + *k*_0_ + *i*_0_ + *α*_2_ − *c*_1_, *e*_1_ + *k*_0_ + *i*_0_ − *c*_1_, and *e*_2_ − *c*_2_, respectively. Under the condition that the profit is high but the cost of time and knowledge is low when sharing knowledge/information, it is concluded that *e*_1_ + *k*_0_ + *i*_0_ + *α*_2_ − *c*_1_ > *e*_1_ + *k*_0_ + *i*_0_ − *c*_1_ > *e*_2_ − *c*_2_; therefore, sharing–sharing is the optimal strategy for ordinary users. However, if the cost of time and knowledge is too high to offset the profit or if a negative benefit occurs, that is, if *e*_2_ − *c*_2_ > *e*_1_ + *k*_0_ + *i*_0_ + *α*_2_ − *c*_1_, then, at this time, nonsharing–nonsharing is the optimal strategy for platform users.

When integrating the common interests of platform operators and users, in order to maximize the profits of game participants and optimize the strategies under different conditions, there are two kinds of results: (1) when sharing knowledge/information, the profit obtained exceeds the cost to be paid, and the game equilibrium point is stabilized in a sharing–sharing strategy. Therefore, both platform operators and users are willing to actively participate in knowledge sharing and spread their own experience so that the platform can gather more flow. (2) If the cost of knowledge/information sharing is high and a loss is suffered, or if it is better not to share knowledge/information, the game equilibrium point is stabilized in a nonsharing–nonsharing strategy; that is, there is a large amount of knowledge and information accumulated in the platform, and users can freely find the desired knowledge on the platform. In this case, most platform members will naturally prefer not to share knowledge.

#### 3.1.3. Evolutionary Game

*(1) Basic Assumptions*. In this evolutionary game model, it is assumed that the platform operators and users have independent but uncertain choices. As time goes by, more and more knowledge/information will be accumulated in the platform, and the coping strategies of users will change according to the content and quality of different platforms. It is assumed that the probability of platform operators choosing the sharing strategy is *m*, and the probability of the platform operators choosing the nonsharing strategy is 1 − *m*; the probability of users choosing the sharing strategy is *n*, and their probability of choosing a non-sharing strategy is 1 − *n*. Therefore, the payoff matrix of the evolutionary game is shown in Table 3.

*(2) Model Analysis*. The above matrix shows that the platform operator can adopt a sharing or a nonsharing strategy. In addition, the expected benefits of the platform operators' sharing strategy are:

(1) $$\begin{array}{c} U_{1m}=n\left(f_{1}+a_{0}+t_{0}+\alpha_{1}-o_{1}\right)+\left(1-n\right)\left(f_{1}+a_{0}+t_{0}-o_{1}\right)=n\alpha_{1}+f_{1}+a_{0}+t_{0}-o_{1}. \end{array}$$

The expected benefits of the platform operators' nonsharing strategy are:

(2) $$\begin{array}{c} U_{2m}=n\left(f_{2}-o_{2}\right)+\left(1-n\right)\left(f_{2}-o_{2}\right)=f_{2}-o_{2}. \end{array}$$

The average expected benefits of the platform operators are:

(3) $$\begin{array}{c} \bar{U_{m}}={mU}_{1m}+\left(1-m\right)U_{2m}=m\left(n\alpha_{1}+f_{1}+a_{0}+t_{0}-o_{1}-f_{2}+o_{2}\right)+f_{2}. \end{array}$$

The strategies that platform users can adopt are sharing or nonsharing. The expected benefits of the platform users' sharing strategy are:

(4) $$\begin{array}{c} U_{1n}=m\left(e_{1}+k_{0}+i_{0}+\alpha_{2}-c_{1}\right)+\left(1-m\right)\left(e_{1}+k_{0}+i_{0}-c_{1}\right)=m\alpha_{2}+e_{1}+k_{0}+i_{0}-c_{1}. \end{array}$$

The expected benefits of the platform users' nonsharing strategy are:

(5) $$\begin{array}{c} U_{2n}=m\left(e_{2}-c_{2}\right)+\left(1-m\right)\left(e_{2}-c_{2}\right)=e_{2}-c_{2}. \end{array}$$

The average expected benefits of the platform users are:

(6) $$\begin{array}{c} \bar{U_{n}}={nU}_{1n}+\left(1-n\right)U_{2n}=n\left(m\alpha_{2}+e_{1}+k_{0}+i_{0}-c_{1}-e_{2}+c_{2}\right)+e_{2}-c_{2}. \end{array}$$

The probability equation for the platform operators' decision on the sharing of knowledge/information is:

(7) $$\begin{array}{c} F\left(m\right)=\frac{dm}{dt}=\left(U_{1m}-\bar{U_{m}}\right)m=m\left(1-m\right)\left(n\alpha_{1}+f_{1}+a_{0}+t_{0}-o_{1}-f_{2}+o_{2}\right). \end{array}$$

When *dm*/*dt* = 0, the derivation shows that the probability of platform operators in choosing knowledge and information sharing decisions is fixed and stable at the equilibrium value. Let us assume *dm*/*dt* = 0. There are three conditions in the solution: *m* = 0, *m* = 1 and *n* = (*f*_2_ + *o*_1_ − *f*_1_ − *o*_2_ − *a*_0_ − *t*_0_)/*α*_1_. At the same time, the three values are the equilibrium points of a replication dynamic equation theory; that is, the probability of the platform operator choosing the knowledge or information sharing strategy will not fluctuate when it reaches these values, but the stability of the three equilibrium points has not yet been judged. According to game theory, due to the evolutionary stability function, it will still return to the equilibrium point, even if the platform operator makes misjudgements or wrong decisions. Thus, the average expected benefits of platform operators are:

(8) $$\begin{array}{c} \bar{U_{n}}={nU}_{1n}+\left(1-n\right)U_{2n}=n\left(m\alpha_{2}+e_{1}+k_{0}+i_{0}-c_{1}-e_{2}+c_{2}\right)+e_{2}-c_{2}. \end{array}$$

Similarly, when the platform user chooses the knowledge/information sharing strategy, the replication dynamic equation of the probability is:

(9) $$\begin{array}{c} F\left(n\right)=\frac{dn}{dt}=\left(U_{1n}-\bar{U_{n}}\right)n=n\left(1-n\right)\left(m\alpha_{2}+e_{1}+k_{0}+i_{0}-c_{1}-e_{1}+c_{2}\right). \end{array}$$

When *dn*/*dt* = 0, the equilibrium solutions of three replication dynamic equations are: *n* = 0, *n* = 1, and *m* = (*e*_2_ − *c*_2_ + *c*_1_ − *e*_1_ − *k*_0_ − *i*_0_)/*α*_2_. This indicates that the probability of platform users choosing knowledge or information sharing strategy tends to be stable when reaching these levels, but the stability of the three equilibrium points cannot be judged. Based on the equilibrium solutions above, it can be seen that the system has five local equilibrium points: (0,0), (0,1), (1,0), (1,1), (((*e*_2_ − *c*_2_ + *c*_1_ − *e*_1_ − *k*_0_ − *i*_0_)/*α*_2_)((*f*_2_ + *o*_1_ − *f*_1_ − *o*_2_ − *a*_0_ − *t*_0_)/*α*_1_)).

In this paper, differential equations are used to describe the probability dynamics of the above two strategies, while the stability of the system evolution is obtained by the Jacobian matrix local stability analysis. The Jacobian determinant matrix is:

(10) $$\begin{array}{c} \left[\begin{array}{cc} \left(1-2m\right)\left(n\alpha_{1}+f_{1}+a_{0}+t_{0}-o_{1}+f_{2}-o_{2}\right) & m\left(1-m\right)\alpha_{1}\\ n\left(1-n\right)\alpha_{2} & \left(1-2n\right)\left(m\alpha_{2}+e_{1}+k_{0}+i_{0}-c_{1}+e_{2}-c_{2}\right) \end{array}\right]. \end{array}$$

The determinant of the matrix is:

(11) $$\begin{array}{c} \left(1-2m\right)\left(n\alpha_{1}+f_{1}+a_{0}+t_{0}-o_{1}+f_{2}-o_{2}\right)*\left(1-2n\right)\left(m\alpha_{2}+e_{1}+k_{0}+i_{0}-c_{1}+e_{2}-c_{2}\right)-m\left(1-m\right)\alpha_{1}*n\left(1-n\right)\alpha_{2}. \end{array}$$

The trace of the determinant is:

(12) $$\begin{array}{c} \left(1-2m\right)\left(n\alpha_{1}+f_{1}+a_{0}+t_{0}-o_{1}+f_{2}-c_{2}\right)+\left(1-2n\right)\left(m\alpha_{2}+e_{1}+k_{0}+i_{0}-c_{1}+e_{2}-c_{2}\right). \end{array}$$

When *n* = *n*^∗^ = (*f*_2_ + *o*_1_ − *f*_1_ − *o*_2_ − *a*_0_ − *t*_0_)/*α*_1_, *dm*/*dt* is 0 all the time, indicating that all values are stable, which means that people with a probability of *m* on the mobile medical information exchange platform will choose to participate in platform knowledge and information sharing; when *m* ≠ (*f*_2_ + *o*_1_ − *f*_1_ − *o*_2_ − *a*_0_ − *t*_0_)/*α*_1_, *m*^∗^ = 0 and *m*^∗^ = 1 are two stable states. When *m* > (*f*_2_ + *o*_1_ − *f*_1_ − *o*_2_ − *a*_0_ − *t*_0_)/*α*_1_, *m*^∗^ = 1 is the evolutionary stability strategy, indicating that the platform is developing well and that the platform operators, the number of which is increasing, are willing to actively share knowledge and information; when *m* < (*f*_2_ + *o*_1_ − *f*_1_ − *o*_2_ − *a*_0_ − *t*_0_)/*α*_1_, *m*^∗^ = 0 is the evolutionary stability strategy; that is, platform operators are unwilling to share knowledge and information on the platform, and the platform vitality is gradually weakened, which finally causes the platform flow to stop increasing or reducing. Similarly, when *m* = *m*^∗^ = (*c*_2_ + *c*_1_ − *e*_1_ − *k*_0_ − *i*_0_ − *e*_2_)/*α*_2_, *dn*/*dt* is 0 throughout, which means that all values are stable; that is, in the platform information exchange stage, users with a probability of *n* will choose not to share but just to browse for knowledge and information; when *m* ≠ (*c*_2_ + *c*_1_ − *e*_1_ − *k*_0_ − *i*_0_ − *e*_2_)/*α*_2_, *n*^∗^ = 0 and *n*^∗^ = 1 are two stable states. In addition, when *m* > (*c*_2_ + *c*_1_ − *e*_1_ − *k*_0_ − *i*_0_ − *e*_2_)/*α*_2_, *n*^∗^ = 1 is the evolutionary stability strategy; that is, platform users will choose knowledge sharing. When *m* < (*c*_2_ + *c*_1_ − *e*_1_ − *k*_0_ − *i*_0_ − *e*_2_)/*α*_2_, *n*^∗^ = 0 is the evolutionary stability strategy; that is, platform users will choose not to share knowledge, as more members of the platform are absorbing knowledge rather than sharing and contributing knowledge.

Combining the process of the one-time game and the evolutionary game, we can see that the equilibrium point will pass through two points, namely, *n*^∗^ = (*f*_2_ + *o*_1_ − *f*_1_ − *o*_2_ − *a*_0_ − *t*_0_)/*α*_1_ and *m*^∗^ = (*c*_2_ + *c*_1_ − *e*_1_ − *k*_0_ − *i*_0_ − *e*_2_)/*α*_2_, and that the whole system will remain stationary at these two stable state points for a period of time. Among the platform operators and users who share knowledge and information at this stage of the mobile medical information exchange platform, the two strategies of sharing and nonsharing will finally stabilize in a sharing–sharing or a nonsharing–nonsharing scenario. Of course, the two results and the selection of the evolutionary path to the equilibrium point are closely related to the game payment matrix and the parameter changes.

#### 3.1.4. Parameter Discussion

*(1) For Platform Operators*. Platform competitiveness improvement is *a*_0_. There are two strategies for platform operators in the information exchange stage of mobile medical platforms, that is, the sharing and nonsharing of knowledge and information. The continuous improvement of platform competitiveness can promote platform operators to share knowledge and information, and the accumulated knowledge of the platform will continue to increase with time. Platform's information capability improvement is *t*_0_. When platform operators share knowledge and information, the platform needs to collect, process, transmit, and service information. During this process, platform's information capability will be improved. Platform's flow improvement is *f*_*i*_. Platform operators share knowledge and information in order to improve the platform flow. At this stage, the platform needs to continuously attract flow and expand the number of platform users, and the ability to do this depends on the operating cost. If the cost is low, platform operators will continue to share knowledge and information.

The knowledge sharing operating cost paid by platform operators is *o*_*i*_. When knowledge and information are shared, platform operators will incur corresponding operating costs, which are greater than the operating costs the operators incur without sharing. The amount of the cost greatly affects knowledge sharing. If the cost of knowledge sharing is too much, platform operators will choose a nonsharing strategy.

For platform users, self-efficacy is *e*_*i*_. Platform users can obtain satisfaction during platform interactions. If there is a strong atmosphere of knowledge exchange and sharing on the platform, the participating users or new users will adapt and participate on the platform as soon as possible and will be willing to share their experiences or knowledge. However, if the knowledge accumulation in a certain field of the platform is close to saturation, the cost of knowledge sharing for users will be higher, and users will be more inclined not to share knowledge; therefore, user activeness will decline.

The improvement of the self-knowledge ability level is *k*_0_. As long as users participate on the platform, they should improve their knowledge regardless of whether or not they share knowledge. The improvement of the knowledge level depends not only on the content digested by users but also on the knowledge reserve provided by the participating platforms. If there are more knowledge reserves, then the wider the scope of the knowledge and the faster the information or knowledge is iteratively updated, the stronger the increase in users' knowledge level or their learning ability. In contrast, the less knowledge reserves there are, the weaker the impact on user's knowledge level and learning ability. Platform identity promotion is *i*_0_. To ensure the identity level, platform users must share information and knowledge. For original entrants, the more frequently knowledge is shared, the greater the value. Therefore, the *i*_0_ of choosing knowledge sharing is greater than the *i*_0_ of not choosing it, and the cost is higher. At this time, users need to decide which choice to adopt according to the benefits. The time and knowledge cost of sharing knowledge and information is *p*_1_. Users participate in the platform to obtain information and knowledge. If the information or knowledge encountered is complex or tacit, the enthusiasm of users to share the information will be greatly reduced because of the great cost of time and knowledge.

### 3.2. Postflow Stage: Mobile Medical Platform

In the postflow stage, the main purpose of the platform is revenue, and the revenue is mainly generated as a result of the content recommendations of platform partners. Considering that platform operators will choose to accept revenue realizable when partners recommend content, the strategy of platform operators is abandoned in the game model of this stage. Generally, platform partners tend to recommend the content of high-flow platforms, and their main appeal is their content promotion ability. Some of the main factors affecting whether users choose to browse the content recommended by platform partners include the form of the content recommendation and the broadcasting behaviour. Users make purchase decisions based on the difference between the psychological price and the platform price. For cooperation in content promotion, platform partners can choose two types of platforms: (1) a high-flow mobile medical platform and (2) a low-flow mobile medical platform. When these different forms of content are pushed to the user, first, the user has the right to choose whether to watch or not to watch. If the watching strategy is chosen, there will be two strategies to choose, that is, to buy or not to buy. In summary, the game relationship between platform partners and end users regarding the selection of a content recommendation can be constructed as shown in Figure 4.

#### 3.2.1. Game between End Users

In view of the online reviews of platform content, the openness and visibility of user feedback, and other reasons, end users can ascertain other users' evaluations of and purchase satisfaction with the end users' preferred content obtained from a mobile medical platform; this information will affect their psychological pricing of the recommendation content.

Accordingly, the following hypotheses are proposed: (1) *p*_1_ is the actual platform price of the recommended content. If both end users buy at the same time, their psychological pricing is *p*_2_. (2) If one does but the other does not, the psychological pricing of the purchased user is *αp*_2_, and the psychological pricing of the nonbuyer is *βp*_2_. (3) When both end users do not buy, their psychological pricing is *γp*_2_. In the process of the purchasing decision, the end user will compare the actual price of the recommendation content with its psychological price and then make the purchasing decision; therefore, *p*_2_ > *αp*_2_ > *p*_1_ > *βp*_2_ > *γp*_2_. The benefit matrix between end users is shown in Table 4.

#### 3.2.2. Game between End Users and Platform Partners

*(1) One-Time Game*. Based on the game between end users and platform partners, this paper proposes the following basic assumptions: the platform partner will pay a fixed cost *c*_1_ for promoting the content of the high-flow platform, the number of content clicks is *n*_1_, and the platform partner will pay *m*_1_ for each click; the platform partner will pay a fixed cost *c*_2_ for promoting content to the low-flow platform, the number of content clicks is *n*_2_, and the platform partner will pay *m*_2_ for each click. Based on the psychological price of end users and their own payment, platform partners need to compare platforms and then make the decision. The partners all expect that high-traffic platforms can bring higher benefits to themselves than other platforms can bring; that is, *n*_1_*r*_2_ − ( *m*_1_*n*_1_ + *c*_1_) > *n*_2_*r*_2_ − ( *m*_2_*n*_2_ + *c*_2_). The revenue matrix of platform partners and end users is shown in Table 5.

#### 3.2.3. Evolutionary Game

Assume that the probability of the “high-flow platform” strategy and the “low-flow platform” strategy is *x* and 1 − *x*, respectively. In addition, when browsing the platform, end users will click and watch according to their favourite content and will abandon the noninterested content; that is, they will choose the nonwatching strategy for the noninterested content. Therefore, it can be assumed that the user chooses “watching” and “nonwatching” strategies, and the two decision probabilities are *y* and 1 − *y*, respectively. The revenue matrix of platform partners and end users is shown in Table 6.

#### 3.2.4. Model Analysis

*(1) Game Relationship between Platform End Users*. First, the game relationship between the end users of the mobile medical platform is analysed. It is assumed that *x*_*i*_ represents the number of neighbours choosing the purchasing strategy. Therefore, the number of neighbours adopting the nonpurchasing strategy is 2 − *x*_*i*_. According to the income matrix, the purchasing income of user *i* at period *t* is *x*_*i*(*t*)_(*p*_2_ − *p*_1_) + (2 − *x*_*i*(*t*)_)(*αp*_2_*p*_1_), and the nonpurchasing income is *x*_*i*(*t*)_(*p*_1_ − *βp*_2_) + (2 − *x*_*i*(*t*)_)(*p*_1_ − *γp*_2_). According to the optimal dynamic response, when *x*_*i*(*t*)_(*p*_2_ − *p*_1_) + (2 − *x*_*i*(*t*)_)(*αp*_2_*p*_1_) > *x*_*i*(*t*)_(*p*_1_ − *βp*_2_) + (2 − *x*_*i*(*t*)_)(*p*_1_ − *γp*_2_), the end user will choose the purchasing strategy. At this time, *x*_*i*(*t*)_ > 2(2p_1_ − *αp*_2_ − *γp*_2_)/(1 − *α* − *γ* + *β*)*p*_2_.When *x*_*i*(*t*)_(*p*_2_ − *p*_1_) + (2 − *x*_*i*(*t*)_)(*αp*_2_*p*_1_) < *x*_*i*(*t*)_(*p*_1_ − *βp*_2_) + (2 − *x*_*i*(*t*)_)(*p*_1_ − *γp*_2_), the end user will choose the nonpurchasing strategy. At this time, *x*_*i*(*t*)_ < 2(2p_1_ − *αp*_2_ − *γp*_2_)/(1 − *α* − *γ* + *β*)*p*_2_.

Considering that platform partners always hope that end users will choose the purchasing strategy all the time, *x*_*i*(*t*)_ > 2(2p_1_ − *αp*_2_ − *γp*_2_)/(1 − *α* − *γ* + *β*)*p*_2_ is the condition that should be satisfied first. Moreover, when *x*_*i*(*t*)_ meets *x*_*i*(*t*)_ ∈ (0, 1], all neighbours adopt the purchasing strategy. After integrating the above two conditions, the final result is as follows: 0 ≤ (2(2p_1_ − *αp*_2_ − *γp*_2_)/(1 − *α* − *γ* + *β*)*p*_2_) < 1. Then, we can obtain the platform pricing range *p*_1_ of the recommendation content by partners. The following solutions are available: ((*α* + *γ*)/2)*p*_2_ ≤ *p*_1_ < ((1 + *α* + *β* + *γ*)/4)*p*_2_. Since *p*_2_ > *αp*_2_ > *p*_1_ > *βp*_2_ > *γp*_2_, it is necessary to determine the platform pricing range of the recommendation content by comparing *αp*_2_ with ((1 + *α* + *β* + *γ*)/4)*p*_2_. When *α* > ((1 + *β* + *γ*)/3), the platform pricing range of the recommendation content is ((*α* + *γ*)/2)*p*_2_ ≤ *p*_1_ < ((1 + *α* + *β* + *γ*)/4)*p*_2_; when *α* < ((1 + *β* + *γ*)/3), the platform pricing range of the recommendation content is ((*α* + *γ*)/2)*p*_2_ ≤ *p*_1_ < *αp*_2_; when *α* = (1 + *β* + *γ*)/3, the platform pricing range of the recommendation content is ((*α* + *γ*)/2)*p*_2_ ≤ *p*_1_ < ((1 + *α* + *β* + *γ*)/4)*p*_2_ = *αp*_2_.

#### 3.2.5. Game Relationship between Platform Partners and End Users

Similar to end users, when choosing platforms, mobile medical platform partners will consider various situations to ensure their benefit maximization and cost minimization. It is assumed that the two probabilities of platform partners choosing “high-flow platform” and “low-flow platform” strategies are denoted by *x* and 1 − *x*, respectively. When browsing on the platform, end users will click and watch according to their favourite content and will abandon the recommendation for content in which they are not interested; that is, they will choose not to watch content in which they are not interested. Therefore, it is assumed that the two probabilities of users choosing “watching” and “nonwatching” strategies are *y* and 1 − *y*, respectively. Platform partners have two available strategies, that is, a “high-flow platform” and a “low-flow platform” strategy, and the expected benefits and average group benefits are as follows:

(13) $$\begin{array}{c} U_{1x}=y\left(n_{1}p_{1}-c_{1}-n_{1}m_{1}\right)+\left(1-y\right)\left(-c_{1}\right)=-c_{1}+n_{1}y\left(p_{1}-m_{1}\right), \end{array}$$

14) $$\begin{array}{c} U_{2x}=y\left(n_{2}p_{1}-c_{2}-n_{2}m_{2}\right)+\left(1-y\right)\left(-c_{2}\right)=-c_{2}+n_{2}y\left(p_{1}-m_{2}\right), \end{array}$$

(15) $$\begin{array}{c} \bar{U_{x}}={xU}_{1x}+\left(1-x\right)U_{2x}=-c_{2}+n_{2}y\left(p_{1}-m_{2}\right)+x\left[c_{2}-c_{1}+n_{1}y\left(p_{1}-m_{1}\right)-n_{2}y\left(p_{1}-m_{2}\right)\right]. \end{array}$$

The expected benefits and the average group benefits of end users choosing “watching” and “nonwatching” strategies are shown below:

(16) $$\begin{array}{c} U_{1y}={xn}_{1}\left(p_{2}-p_{1}\right)+\left(1-x\right)n_{2}\left(p_{2}-p_{1}\right)=\left(p_{2}-p_{1}\right)\left[n_{2}+\left(n_{1}-n_{2}\right)x\right],\\ U_{2y}=x*0+\left(1-x\right)*0=0\;\bar{U_{y}}={yU}_{1y}+\left(1-y\right)U_{2y}=\left(p_{2}-p_{1}\right)\left[n_{2}+\left(n_{1}-n_{2}\right)x\right]y. \end{array}$$

The replication dynamic equation of platform partners choosing the “high-flow network platform” strategy is:

(17) $$\begin{array}{c} F\left(x\right)=\frac{dx}{dt}=x\left(U_{1x}-\bar{U_{x}}\right)=x\left(1-x\right)\left[\left(c_{2}-c_{1}\right)+n_{1}y\left(p_{1}-m_{1}\right)-n_{2}y\left(p_{1}-m_{2}\right)\right]. \end{array}$$

The replication dynamic equation of the end user choosing the “watching” strategy is:

(18) $$\begin{array}{c} F\left(y\right)=\frac{dy}{dt}=y\left(U_{1y}-\bar{U_{y}}\right)=y\left(1-y\right)\left(c_{2}-c_{1}\right)\left[n_{2}+\left(n_{1}-n_{2}\right)x\right]. \end{array}$$

The matrix of the Jacobian determinant is:

(19) $$\begin{array}{c} J=\left[\begin{array}{cc} \left(1-2x\right)\left[\left(c_{2}-c_{1}\right)+n_{1}y\left(p_{1}-m_{1}\right)-n_{2}y\left(p_{1}-m_{2}\right)\right] & x\left(1-x\right)\left[n_{1}\left(p_{1}-m_{1}\right)-n_{2}\left(p_{1}-m_{2}\right)\right]\\ y\left(1-y\right)\left(p_{2}-p_{1}\right)\left(n_{1}-n_{2}\right) & \left(1-2y\right)\left(p_{2}-p_{1}\right)\left[n_{2}+\left(n_{1}-n_{2}\right)x\right] \end{array}\right]. \end{array}$$

The trace of determinant is:

(20) $$\begin{array}{c} \left(1-2x\right)\left[\left(c_{2}-c_{1}\right)+n_{1}y\left(p_{1}-m_{1}\right)-n_{2}y\left(p_{1}-m_{2}\right)\right]+\left(1-2y\right)\left(p_{2}-p_{1}\right)\left[n_{2}+\left(n_{1}-n_{2}\right)x\right]. \end{array}$$

It can be seen from the above two equations that the Jacobi determinant has four equilibrium points, namely, (0, 0), (0, 1), (1, 0), and (1, 1). Considering that this model aims to find the stability strategy for the best interests of platform partners, it is necessary only to judge the two strategies (0,1) and (1,1) in which the end user watches. When the stability strategy is (0,1), the value of the determinant is ‐(*p*_2_ − *p*_1_)[(*c*_2_ − *c*_1_) + *n*_1_(*p*_1_ − *m*_1_) − *n*_2_(*p*_1_ − *m*_2_)]*n*_2_ > 0, and the trace is (*c*_2_ − *c*_1_) + *n*_1_(*p*_1_ − *m*_1_) − *n*_2_(*p*_1_ − *m*_2_) − (*p*_2_ − *p*_1_)*n*_2_ < 0; then, we obtain *p*_1_ < (−(*c*_2_ − *c*_1_) + *m*_1_*n*_1_ − *m*_2_*n*_2_ + *p*_2_*n*_2_)/*n*_1_. When the stability strategy is (1,1), the value of the determinant is (*p*_2_ − *p*_1_)[(*c*_2_ − *c*_1_) + *n*_1_(*p*_1_ − *m*_1_) − *n*_2_(*p*_1_ − *m*_2_)]*n*_1_ > 0, and the trace is −[(*c*_2_ − *c*_1_) + *n*_1_(*p*_1_ − *m*_1_) − *n*_2_(*p*_1_ − *m*_2_)] − (*p*_2_ − *p*_1_)*n*_1_ < 0; then, we obtain *p*_1_ > (*m*_1_*n*_1_ − *m*_2_*n*_2_ − (*c*_2_ − *c*_1_))/(*n*_1_ − *n*_2_).

#### 3.2.6. Comprehensive Analysis of Game Relations

A comprehensive analysis of the above two game models can be summarized by the following two cases, and the corresponding conclusions are drawn as follows: in the first case, the platform partners cooperate with high-flow mobile medical platforms and promote content for the high-flow platforms. When *α* > (1 + *β* + *γ*)/3, the platform pricing of recommendation content meets conditions ((*α* + *γ*)/2)*p*_2_ ≤ *p*_1_ < ((1 + *α* + *β* + *γ*)/4)*p*_2_ and *p*_1_ > (*m*_1_*n*_1_ − *m*_2_*n*_2_ − (*c*_2_ − *c*_1_))/(*n*_1_ − *n*_2_); when *α* > (1 + *β* + *γ*)/3, the platform pricing of recommendation content meets conditions ((*α* + *γ*)/2)*p*_2_ ≤ *p*_1_ < *αp*_2_ and *p*_1_ > (*m*_1_*n*_1_ − *m*_2_*n*_2_ − (*c*_2_ − *c*_1_))/(*n*_1_ − *n*_2_). When *α* > (1 + *β* + *γ*)/3, the platform pricing of recommendation content meets conditions ((*α* + *γ*)/2)*p*_2_ ≤ *p*_1_ < ((1 + *α* + *β* + *γ*)/4)*p*_2_ = *αp*_2_ and *p*_1_ > (*m*_1_*n*_1_ − *m*_2_*n*_2_ − (*c*_2_ − *c*_1_))/(*n*_1_ − *n*_2_). In the second case, the platform partners cooperate with low-flow mobile medical platforms to promote content on low-flow platforms. When *α* > (1 + *β* + *γ*)/3, the platform pricing of recommendation content meets conditions ((*α* + *γ*)/2)*p*_2_ ≤ *p*_1_ < ((1 + *α* + *β* + *γ*)/4)*p*_2_ and *p*_1_ < (−(*c*_2_ − *c*_1_) + *m*_1_*n*_1_ − *m*_2_*n*_2_ + *p*_2_*n*_2_)/*n*_1_; when *α* > (1 + *β* + *γ*)/3, the platform pricing of recommendation content meets conditions ((*α* + *γ*)/2)*p*_2_ ≤ *p*_1_ < *αp*_2_ and *p*_1_ < (−(*c*_2_ − *c*_1_) + *m*_1_*n*_1_ − *m*_2_*n*_2_ + *p*_2_*n*_2_)/*n*_1_. When *α* > (1 + *β* + *γ*)/3, the platform pricing of recommendation content meets conditions ((*α* + *γ*)/2)*p*_2_ ≤ *p*_1_ < ((1 + *α* + *β* + *γ*)/4)*p*_2_ = *αp*_2_ and *p*_1_ < (−(*c*_2_ − *c*_1_) + *m*_1_*n*_1_ − *m*_2_*n*_2_ + *p*_2_*n*_2_)/*n*_1_.

## 4. Simulation

When browsing the content recommended by the platform partner, the end user will develop a psychological price judgement of the interested content and compare the platform price with it to decide whether to buy or not. Therefore, the platform price of content recommended by the platform partner will be affected by the psychological pricing coefficient of the end user for the recommendation content. In the following two cases, we analyse the influence of the psychological pricing coefficient *β* on the platform selling price of recommendation content *p*_1_. Combined with the current development status of a mobile medical platform, the simulation parameters are selected according to the selling price of the content recommended by the platform partners of current typical platforms. Referring to other research literatures about the parameter settings of the customer psychological pricing coefficient, the parameter values are determined.

In the first case, when *γ* is given and *α* = 1 + *β* + *γ*/3, the influence of *β* on *p*_1_ is analysed. Assuming *γ* = 0.100 and *p*_2_ = 50, we analyse the change of *p*_1_ when *β* changes from 0.1 to 0.54.

As shown in Figure 5, when *γ* is given and *α* = 1 + *β* + *γ*/3, the platform price of recommendation content will increase as *β* increases, and the pricing range will gradually increase. The relevance of the above results to the management practice of mobile medical platforms is that once the platform partners obtain the desired content and can determine the acceptable psychological price of the target users in some way, they can make the appropriate pricing adjustments. At the same time, to develop precise marketing strategies, the platform partners can also track, analyse, and utilize the information of recent users on mobile medical platforms. The psychological price of end users for the recommendation content can be improved in a reasonable way. For example, the platform partner can appropriately boost the publicity quality of the content and the accuracy of the directional broadcast, which will greatly increase the platform price of the recommendation content. Meanwhile, they can also carry out different price combinations in different periods to generate a win-win profit and brand situation.

In the second case, given *α*_,_*γ*_,_ and that the size of the relationship between *α* and 1 + *β* + *γ*/3 is uncertain, the effect of *β* on *p*_1_ is analysed. Assuming *α* = 0.5, *γ* = 0.1, and *p*_2_ = 100, when *β* changes from 0.1 to 0.5, the change of *p*_1_ is shown in Figure 6. When *α*, *γ* is given, and the size relationship between *α* and 1 + *β* + *γ*/3 is uncertain, as *β* increases, the price range of the commodity increases first, then remains unchanged; in this case, the lower price limit does not change, and the upper limit increases first and remains invariant; that is, when *β* = 0.401, the change of *β* exerts no effect on the network price.

The above results reveal that improving the publicity quality of the recommendation content can improve the psychological price of the product of the end user that might otherwise choose a nonpurchasing strategy and is helpful for the platform partner in enabling the partner to raise the price of the content. The influencing factors among users are different and difficult to judge, and the orientation accuracy of the recommendation content will be affected; therefore, it may not be possible to always increase the platform price, as there may be some end users who will not purchase after the price reaches a certain level. Therefore, unlike the first case, the range of the pricing strategy adjustment of platform partners will be limited.

Platform partners should work closely with the mobile medical platform to obtain the desired effective information on purchasing behaviour from the platform and should maximize the utility of this information. Otherwise, blindly putting on content or just increasing the number of referrals may not stimulate reluctant purchasing users to engage in purchase behaviour and may ultimately fail to achieve the goal of increasing the expected returns.

In conclusion, through the continuous game and strategy selection of platform operators, platform partners, and end users, we can promote the increase of platform revenue and then realize the dynamic equilibrium of the three interests at the core layer in the mobile medical platform business ecosystem and promote the stable and healthy development of the platform.

## 5. Implications on the Support Strategy of Mobile Medical Platform Business Ecosystem

### 5.1. Support Strategy at Preflow Stage

#### 5.1.1. Promotion Strategy for Platform Operators

Increase platform inclusiveness, and build knowledge bases in different fields.

Platform operators need to continuously support knowledge and information sharing, while sorting out and classifying all kinds of knowledge, establishing knowledge bases in different fields, strengthening the knowledge linkage between platforms and users, and eliminating the knowledge generation gap.

Implement flat management, and respond in a timely manner to issues of high concern.

The platform should develop a flat organizational structure, reduce information barriers, improve the information processing capabilities of the platform, and create more value in different knowledge chains. At the same time, the platform should be able to respond in a timely manner to issues of high concern so that users are willing to participate in activities and to remain in touch with the platform.

Enhance policy support, and build (building) a good (excellent) platform service system.

The government should introduce relevant supporting policies or regulations, such as multisite physician practice and “Internet + medical” policies, to guide capital and resources into the mobile medical field. At the same time, laying a solid foundation for the construction of a good ecosystem of the platform, the government should actively encourage financial institutions, investment institutions, legal institutions, and other intermediary agencies to enter the platform.

### 5.2. Incentives and Safeguards for Platform Users

Strengthen knowledge protection, and mine knowledge needs.

Appropriate knowledge protection measures should be developed to provide the sharers with a sense of security and to thereby attract more users or consumers to participate in knowledge sharing on the platform. Simultaneously, to meet the internal needs of platform users, the enthusiasm of users to share knowledge should be fully mobilized.

Implement incentives to improve platform activity.

Through commendations of honour, material reward, and other forms of rewards, the sense of participation of users can be stimulated to form an overall relationship between users and platforms. Paying close attention to the development of the platform and stimulating platform's use by more users can improve platform's activity and increase the platform flow.

Guarantee the quality of knowledge sharing, and enhance the professionalism of the platform.

Efforts should be made to control the content of knowledge sharing and to guide it as much as possible toward high-quality medical knowledge. At the same time, the ability to identify shared knowledge should be improved, content irrelevant to the characteristics of the platform should be deleted in a timely manner, a good quality system of knowledge sharing should be built, and the professionalism of the platform should be enhanced.

### 5.3. Support Strategy at Postflow Stage

#### 5.3.1. Support for Platform Operators

Improve the operating capacity of platform operators.

Artificial intelligence, big data, cloud computing, and other technologies should be integrated and applied to fully exploit the relationship between various types of information, and platform operating costs should be reduced, thereby cutting down the cost of platform partners and increasing the enthusiasm of platform partners.

Create a good external environment.

To guide and promote the development of the platform, the government should take measures, such as introducing policies to accelerate the interconnection of medical information, promoting the establishment of electronic health records, and encouraging investment institutions to invest in mobile medical platforms. In addition, to make the professional quality of the platform more prominent, third-party service institutions should be invited to provide consultancy, academic research, project supervision, and other services for the platform.

Introduce commercial insurance to balance the interests of all parties.

Commercial insurance with a fee control mechanism should be introduced to coordinate and balance the interests between platform operators and users. At the same time, to stimulate the sustainable development of the mobile medical platform, the fee control mechanism of medical insurance should be improved, the medical service process should be effectively supervised, and the dynamic balance of interests among users, platform partners, and platforms should be promoted.

#### 5.3.2. Support for Platform Partners

Give play to the incentive and supervisory role of the platform.

To motivate platform partners to increase content recommendation, the cost of content promotion and click payments should be reduced, and recommendation subsidies should be provided. At the same time, to ensure that the quality and quantity of platform's content are simultaneously improved, the platform should strengthen the supervision and the monitoring of the contents recommended by partners.

Deepen data resource cooperation of the platform.

Through premarket surveys, platform partners can understand the maximum affordable psychological price of end users for their recommended content and the degree of interaction between end users in terms of purchasing psychology and behaviour. At the same time, to track and analyse users' needs and to conduct precise marketing strategies, platform partners should strengthen their cooperation with platform operators, making full use of the consumption and preference data resources of platform users.

Strengthen the propaganda quality of platform partners.

By appropriately increasing the recommendation quality of product's online content and the accuracy of the directional promotion, the platform partners can increase the psychological price of end users who are reluctant to purchase the recommendation content; this pricing flexibility will enable the platform price range of the promotional content to expand, thereby providing more space for different price combinations at different times and achieving a win-win situation for both profit and the brand.

#### 5.3.3. Support for End Users

Encourage end users to participate in content consumption.

By reducing the cost of obtaining information, such as costs related to time and energy, the content clicking and points sharing system, the lifelong free use of identity, and to other measures, the platform can attract end users to continuously interact and consume content on the platform.

Strengthen the quality of knowledge sharing and content promotion.

The platform should promote deeper and broader information sharing, provide better services for end users in order to attract platform users, and provide users with more incentives to identify with the platform. Platform partners should provide more accurate content recommendations based on users' needs, improve the psychological pricing of users' content, and encourage users to continuously participate in platform activities.

## 6. Conclusions and Prospect

### 6.1. Conclusions

By analysing the game revenue matrix and replication dynamic equations of platform operators, platform partners, and end users and through conducting multiple iterative evolution games, this paper obtains the dynamic equilibrium strategy of the interests of the three parties participating in the mobile medical platform in the preflow period and the postflow period.

In the preflow period, with the platform knowledge sharing behaviour as the object, the following three supporting strategies for platform operators are proposed: (1) increase platform inclusiveness and build knowledge bases in different fields; (2) implement flat management and develop timely responses to issues of high concern; and (3) enhance policy support and build an efficient platform service system. Additionally, the following three supporting strategies for platform users are also presented: (1) strengthen knowledge protection and mine knowledge needs; (2) implement incentives to facilitate platform activity; and (3) guarantee the quality of knowledge sharing and enhance the professionalism of the platform. In this way, the knowledge sharing of the mobile medical platform can be encouraged and guaranteed, and more users can be attracted to participate; therefore, the platform flow can be enhanced.

In the postflow period, the crucial issues are flow stimulation and revenue creation. Solving these issues will then help to build a dynamic interest balancing point among platform operators, platform partners, and end users, thereby facilitating the realization of platform's evolution. Three strategies are proposed: (1) supporting platform operator and including the strengthening of the operations capability of the platform operators, creating a good external environment, and introducing commercial insurance to balance the interests of all parties; (2) supporting platform partners, strategies proposed to enhance the motivation, and supervision role of the platform, deepen the cooperation of platform data resources, and strengthen the publicity quality of the platform partners; and (3) supporting end users, strategies that encourage them to participate in content consumption and that strengthen the mutual linkage between knowledge sharing and content recommendation quality.

### 6.2. Limitation and Prospect

Based on the related literature review and comprehensive use of a game model, simulation, and other methods, providing references for further research, this paper conducts a detailed study on a mobile medical platform business ecosystem. However, due to the limits of research time and capability, there are still some areas needing further improvement: (1) in choosing the factors of the two-stage dynamic equilibrium of the interests of a mobile medical platform business ecosystem, only the core layer is considered, while the influence of the peripheral layer is not considered. This leads to a limitation of the conclusion. In future research, the influence factors of the peripheral layer can be introduced, and the incentive mechanism can be set up. (2) From the perspective of research methods, this paper sets up data and conducts a simulation according to the platform theory, which will inevitably reduce the validity of the research. Therefore, for future studies, data should be set up according to the characteristics of the mobile medical platform. Meanwhile, more methods such as quantitative measurement and cases study should be comprehensively adopted to conduct research. (3) Based on this theoretical study, for the proposal of better countermeasures and policy suggestions, future research can adopt a field study approach to track the actual platform operations.

## Figures and Tables

**Figure 1:** Platform business ecosystem model.

**Figure 2:** Business ecosystem model of mobile medical platform.

**Figure 3:** Three-dimensional structure model of a mobile medical platform business ecosystem.

**Figure 4:** The game between the platform partners and the end users.

**Figure 5:** Comparison of psychological pricing and platform price.

**Figure 6:** Comparison of psychological pricing and platform price.

**Table 1:** Parameter description.

Parameter	Description
*f*_1_	The increase of platform flow when the platform operator chooses the sharing knowledge/information strategy
*a*_0_	The improvement of platform competitiveness when the platform operator chooses the sharing knowledge/information strategy
*t*_0_	The improvement of platform information capability when the platform operator chooses the sharing knowledge/information strategy
*o*_1_	The operating cost when the platform operator chooses the sharing knowledge/information strategy
*f*_2_	The increase of platform flow when the platform operator chooses the nonsharing knowledge/information strategy
*o*_2_	The operating cost when the platform operator chooses the nonsharing knowledge/information strategy
*e*_1_	The improvement of self-efficacy when the platform user chooses the sharing knowledge/information strategy
*k*_0_	The improvement of knowledge capability when the platform user chooses the sharing knowledge/information strategy
*i*_0_	The improvement of platform identity when the platform user chooses the sharing knowledge/information strategy
*c*_1_	The knowledge cost and time when the platform user chooses the sharing knowledge/information strategy
*e*_2_	The improvement of self-efficacy when the platform user chooses the nonsharing knowledge/information strategy
*c*_2_	The time cost when the platform user chooses the nonsharing knowledge/information strategy
*α*_1_	The extra benefit of the platform when both parties choose the sharing knowledge/information strategy
*α*_2_	The extra benefit of the platform users when both parties choose the sharing knowledge/information strategy

**Table 2:** Game payment matrix.

Platform operator	Platform user	
	Sharing	Nonsharing
Sharing	*f*_1_ + *a*_0_ + *t*_0_ + *α*_1_ − *o*_1_, *e*_1_ + *k*_0_ + *i*_0_ + *α*_2_ − *c*_1_	*f*_1_ + *a*_0_ + *t*_0_ − *o*_1_, *e*_2_ − *c*_2_
Nonsharing	*f*_2_ − *o*_2_, *e*_1_ + *k*_0_ + *i*_0_ − *c*_1_	*f*_2_ − *o*_2_, *e*_2_ − *c*_2_

**Table 3:** Evolutionary game return matrix.

Platform operator	Platform user	
	Sharing	Nonsharing
Sharing	*m*(*f*_1_ + *a*_0_ + *t*_0_ + *α*_1_ − *o*_1_), *n*(*e*_1_ + *k*_0_ + *i*_0_ + *α*_2_ − *c*_1_)	*m*(*f*_1_ + *a*_0_ + *t*_0_ − *o*_1_), (1 − *n*)(*e*_2_ − *c*_2_)
Nonsharing	(1 − *m*)(*f*_2_ − *o*_2_), *n*(*e*_1_ + *k*_0_ + *i*_0_ − *c*_1_)	(1 − *m*)(*f*_2_ − *o*_2_), (1 − *n*)(*e*_2_ − *c*_2_)

**Table 4:** Income matrix between end users.

End user 2	End user 1	
	Purchasing	Nonpurchasing
Purchasing	*p*_2_ − *p*_1_, *p*_2_ − *p*_1_	*αp*_2_ − *p*_1_, *p*_1_ − *βp*_2_
Nonpurchasing	*p*_1_ − *βp*_2_, *βp*_2_ − *p*_1_	*p*_1_ − *γp*_2_, *p*_1_ − *γp*_2_

**Table 5:** Revenue matrix of platform partners and end users.

Platform operator	End user	
	Watching	Nonwatching
High-flow platform	*n*_1_ *p*_1_ − *c*_1_ − *n*_1_*m*_1_, *n*_1_*p*_1_ − *c*_1_ − *n*_1_*m*_1_, *n*_1_(*p*_2_ − *p*_1_)	−*c*_1_, 0
Low-flow platform	*n*_2_ *p*_1_ − *c*_2_ − *n*_2_*m*_2_, *n*_2_(*p*_2_ − *p*_1_)	−*c*_2_, 0

**Table 6:** Evolutionary game matrix.

Platform operator	End user	
	Watching	Nonwatching
High-flow platform	*x*(*n*_1_*p*_1_ − *c*_1_ − *n*_1_*m*_1_), *y*(*n*_1_(*p*_2_ − *p*_1_))	−*xc*_1_, 0
Low-flow platform	(1 − *x*)(*n*_2_*p*_1_ − *c*_2_ − *n*_2_*m*_2_), *y*(*n*_2_(*p*_2_ − *p*_1_))	−(1 − *x*)*c*_2_, 0

## Data Availability

The data used to support the findings of this study are included within the article.
